# Programmed NP Cell Death Induced by Mitochondrial ROS in a One-Strike Loading Disc Degeneration Organ Culture Model

**DOI:** 10.1155/2021/5608133

**Published:** 2021-08-31

**Authors:** Bao-Liang Li, Xizhe Liu, Manman Gao, Fu Zhang, Xu Chen, Zhongyuan He, Jianmin Wang, Wei Tian, Dafu Chen, Zhiyu Zhou, Shaoyu Liu

**Affiliations:** ^1^Innovation Platform of Regeneration and Repair of Spinal Cord and Nerve Injury, Department of Orthopaedic Surgery, The Seventh Affiliated Hospital, Sun Yat-sen University, Shenzhen 518107, China; ^2^Guangdong Provincial Key Laboratory of Orthopedics and Traumatology, Orthopaedic Research Institute/Department of Spinal Surgery, The First Affiliated Hospital of Sun Yat-sen University, Guangzhou 510080, China; ^3^Department of Sport Medicine, Inst Translat Med, The First Affiliated Hospital of Shenzhen University, Shenzhen Second People's Hospital, Shenzhen 518000, China; ^4^Guangdong Key Laboratory for Biomedical Measurements and Ultrasound Imaging, School of Biomedical Engineering, Shenzhen University Health Science Center, Shenzhen 518060, China; ^5^Laboratory of Bone Tissue Engineering, Beijing Laboratory of Biomedical Materials, Beijing Research Institute of Orthopaedics and Traumatology, Beijing Jishuitan Hospital, Beijing 100035, China

## Abstract

Increasing evidence has indicated that mitochondrial reactive oxygen species (ROS) play critical roles in mechanical stress-induced lumbar degenerative disc disease (DDD). However, the detailed underlying pathological mechanism needs further investigation. In this study, we utilized a one-strike loading disc degeneration organ culture model to explore the responses of intervertebral discs (IVDs) to mechanical stress. IVDs were subjected to a strain of 40% of the disc height for one second and then cultured under physiological loading. Mitoquinone mesylate (MitoQ) or other inhibitors were injected into the IVDs. IVDs subjected to only physiological loading culture were used as controls. Mitochondrial membrane potential was significantly depressed immediately after mechanical stress (*P* < 0.01). The percentage of ROS-positive cells significantly increased in the first 12 hours after mechanical stress and then declined to a low level by 48 hours. Pretreatment with MitoQ or rotenone significantly decreased the proportion of ROS-positive cells (*P* < 0.01). Nucleus pulposus (NP) cell viability was sharply reduced at 12 hours after mechanical stress and reached a stable status by 48 hours. While the levels of necroptosis- and apoptosis-related markers were significantly increased at 12 hours after mechanical stress, no significant changes were observed at day 7. Pretreatment with MitoQ increased NP cell viability and alleviated the marker changes by 12 hours after mechanical stress. Elevated mitochondrial ROS levels were also related to extracellular matrix (ECM) degeneration signs, including catabolic marker upregulation, anabolic marker downregulation, increased glycosaminoglycan (GAG) loss, IVD dynamic compressive stiffness reduction, and morphological degradation changes at the early time points after mechanical stress. Pretreatment with MitoQ alleviated some of these degenerative changes by 12 hours after mechanical stress. These changes were eliminated by day 7. Taken together, our findings demonstrate that mitochondrial ROS act as important regulators of programmed NP cell death and ECM degeneration in IVDs at early time points after mechanical stress.

## 1. Introduction

Degenerative disc disease (DDD) is a chronic spinal disorder characterized by structural failure of the intervertebral disc (IVD), increased proteolytic activity, nucleus pulposus (NP) cell death, and proinflammatory cytokine release [1, 2]. Lumbar DDD is one of the most common chronic degenerative diseases worldwide. It impacts forty percent of people aged 40 years and affects more than eighty percent of the population aged 80 years, with nearly twenty percent of people with lumbar DDD showing a poor response to nonsurgical treatment [3]. Hence, there is an urgent need for a deep understanding of the underlying molecular mechanisms responsible for DDD for the sake of better management.

Nonphysiological mechanical stress (MS) is viewed as a significant risk factor for the development of lumbar DDD [4]. Excessive MS results in cell death and extracellular matrix (ECM) degradation, which leads to significant structural changes in IVDs [5]. Necroptosis and apoptosis are the two principal types of programmed cell death that have been implicated in lumbar DDD [6, 7]. Despite mounting evidence, the mechanisms underlying MS-induced DDD have not been fully elucidated.

Mitochondria are central cytoplasmic hubs essential for not only cellular metabolism but also various types of programmed cell death, including apoptosis and necroptosis, due to their production of reactive oxygen species (ROS) and other prodeath mediators [8]. Multiple complex mechanisms underlie MS-induced mitochondrial ROS production, including intracellular Ca^2+^ overload and cytoskeletal strain [9–11]. It was recently demonstrated that mechanical stimulation induces the endoplasmic reticulum Ca^2+^ releases and extracellular Ca^2+^ influx [12]. Excessive cytosolic Ca^2+^ elevations induce mitochondrial depolarization and ROS generation [13]. As the cytoskeleton interacts heavily with mitochondria, it is not surprising that cell strain results in mitochondrial strain and ROS generation. In addition, dissolution of the cytoskeleton by reagents prevents impact-induced ROS generation [9].

Several studies have emphasized the importance of mitochondrial ROS in NP cell mechanical injury. Excessive ROS generation activates multiple apoptosis pathways by causing damage to proteins, nucleic acids, lipids, membranes, and organelles. Mitochondrial-derived oxidative stress is thought to contribute to the necroptotic pathway at the receptor-interacting protein kinase 3 (RIPK3) or mixed-lineage kinase domain-like protein (MLKL) level [14]. A recent study has reported that mitochondrial ROS promote RIPK1 autophosphorylation on serine residue 161 (S161) and then recruit RIPK3 to further form a functional necrosome and that necrosomal RIPK3 enhances ROS production [8]. In recent years, a growing number of research articles have highlighted the critical role of mitochondrial ROS in the programmed death of NP cells, providing crucial novel insights into the progression of lumbar DDD [15]. For example, a study on isolated NP cells indicated that increased RIPK1 expression following compression-induced injury induces mitochondrial dysfunction and oxidative stress. However, how mitochondrial ROS affect NP cell viability in IVDs is still unclear.

Enhanced expression of catabolic markers such as matrix metalloproteases (MMPs) and a disintegrin and metalloproteinase with thrombospondin motif (ADAMTS) proteins and loss of glycosaminoglycan have been observed in NP tissue after MS. Interestingly, Nasto et al. reported that mitochondrial ROS induce MMP gene expression in NP cells in vitro, suggesting that mitochondrial ROS plays a pathological role in aging-related IVD degeneration [16]. Several other reports have demonstrated that antioxidative therapy suppresses the gene expression of ECM-destructive enzymes in cartilage after MS [17]. Therefore, we hypothesized that MS-induced catabolic marker expression and ECM degeneration are partly mediated by mitochondrial ROS.

Several studies have shown that high-impact loading is a significant factor contributing to DDD [18–24]. Based on this finding, we successfully established a disc degeneration organ culture model via one-strike loading [24]. This model showed signs of early degeneration, including annulus fibrosus (AF) fissures, ECM degradation, glycosaminoglycan (GAG) release, and upregulated catabolic marker gene expression. Our one-strike loading model may not fully reveal the whole process of DDD development. Nevertheless, it is well suited for investigating the pathogenesis of MS-induced DDD at the early stage.

The objective of the present study was to investigate the occurrence of programmed cell death, ECM degeneration, and mitochondrial ROS production after MS in a one-strike loading model. More importantly, the correlations among MS, mitochondrial ROS, programmed cell death, and ECM degeneration were evaluated by measuring cellular reactions to help elucidate the molecular pathophysiology of DDD.

## 2. Materials and Methods

### 2.1. Isolation and Cultivation of IVDs

Tails from bovines were obtained from a local abattoir. As we used leftovers of the slaughterhouse, no approval of an ethical committee was required according to Chinese regulations. IVD isolation and cultivation were carried out as previously described on day 0 [19]. In brief, after dissecting the surrounding soft tissue, individual IVDs with endplates were resected with a band saw. The endplates were rinsed with phosphate-buffered saline (PBS) using an APEXPULSE Disposable Pulse Lavage system (Apex, Guangzhou, China). Then, the IVDs were washed with PBS containing 10% penicillin/streptomycin (Gibco, Waltham, MA) for 15 minutes on a shaking table. The IVDs were then incubated with Dulbecco's modified Eagle's medium (DMEM, Sigma-Aldrich, Munich, Germany) supplemented with 2% fetal calf serum (FCS), 1% penicillin/streptomycin, 1% ITS+1 (Sigma-Aldrich), 50 *μ*g/ml L-ascorbic acid (Sigma-Aldrich), and 0.1% Primocin (InvivoGen, San Diego, CA, USA) in a humidified (85%) atmosphere with 5% CO_2_ at 37°C. All IVDs were cultured under physiological loading (0.02–0.2 MPa; 0.2 Hz; 1 hour/day) within a custom-designed bioreactor from day 1 (Figure 1(a)). The culture medium was replaced once a day after physiological loading. IVDs from the same tail were randomly assigned to different groups. IVDs subjected to only physiological loading culture were assigned to control (CON) groups.

### 2.2. Mechanical Stress

IVDs were subjected to MS using a custom-made universal mechanical tester in a custom-designed incubation chamber at room temperature on day 1 (Figure 1(a)). During the MS period, the IVDs were incubated in a culture medium to prevent dehydration. The IVDs were first subjected to a preload of 10 N for 3 minutes to prevent overhydration and to ensure reliable contact between the endplate, the incubation chamber, and the mechanical tester. MS injury was applied for one second with a strain of 40% of the disc height. Following MS injury, the IVDs were analyzed or incubated in a culture medium with daily physiological loading for another 1 to 7 days.

### 2.3. Dynamic Compressive Stiffness

The dynamic compressive stiffness was gauged by the custom-designed bioreactor at several time points: on day 1, day 2, and day 7 after overnight free-swelling culture [25]. The discs were first preloaded with 10% strain for 3 minutes and then loaded with 10 rounds of sinusoidal compression at 5–15% strain. Dynamic stress was determined by the following equation: (*F*_max_–*F*_min_)/*S*. *F*_max_ and *F*_min_ represent the maximum and minimum forces achieved during one round, respectively, and *S* is the sectional area of the IVD. The dynamic compressive stiffness was gauged for every loading round, and the average value from 10 rounds was calculated. The stiffness gauged on day 1 was used as a baseline for standardization.

### 2.4. Inhibitor Studies

For inhibitor studies, various reagents were dissolved in dimethyl sulfoxide (DMSO) and diluted in PBS. Then, 100 *μ*l of PBS containing reagent was injected into the NP tissue with a 26-gauge needle during the middle of the dynamic loading cycle. To exclude potential interference, 100 *μ*l of PBS containing 0.05% DMSO was injected into CON IVDs. After 2 hours of free-swelling recovery, the IVDs were subjected to a one-time MS injury. To distinguish between apoptosis and necroptosis, the RIPK1 inhibitor necrostatin-1 (Nec-1, 80 *μ*m, MCE, NJ, USA) and the pan-caspase inhibitor N-benzyloxycarbonyl-Val-Ala-Asp-fluoromethylketone (Z-VAD-FMK, 50 *μ*m, MCE) were used. The electron transport chain inhibitor rotenone (20 *μ*m, Sigma-Aldrich) was used to inhibit mitochondrial ROS generation. To verify the involvement of mitochondrial ROS in MS-induced programmed NP cell death and disc degeneration, the mitochondrial ROS scavenger mitoquinone mesylate (MitoQ, 4 *μ*m, MCE) was used. MitoQ was mixed into the culture medium after daily medium renewal.

### 2.5. Cell Viability Assay

Cell viability was evaluated using calcein acetoxymethyl ester (calcein AM, eBioscience, Frankfurt, Germany) and propidium iodide (PI, MCE). In this system, green fluorescence indicates viable cells with intact membranes, green/red fluorescence indicates viable cells with compromised plasma membranes, and red fluorescence indicates dead cells [26]. For histological analysis, the AF and endplates were dissected with a scalpel. NP tissue was cut into slices (100 *μ*m) with a vibrating microtome (Leica VT1200S, Leica Microsystems, Germany). The NP tissue slices were incubated with a culture medium containing 1 *μ*g/ml calcein AM and 1 *μ*g/ml PI for one hour at 37°C. After washing with PBS, the slices were immediately viewed using an inverted confocal laser scanning microscope (Zeiss Confocal LSM 780, Carl Zeiss Jena GmbH, Jena, Germany), and one random image per disc was analyzed. The numbers of viable and dead cells were measured manually using ImageJ software (National Institutes of Health, USA).

### 2.6. Measurement of Mitochondrial Membrane Potential

Mitochondrial membrane potential was evaluated using 5,5′,6,6′-tetrachloro-1,1′,3,3′-tetraethylbenzimidazolocarbocyanine iodide (JC-1, MCE). In cells with normal mitochondria, JC-1 aggregates in mitochondria with a high red/green fluorescence intensity ratio. In cells with compromised mitochondria, JC-1 aggregates become JC-1 monomers, and the red/green fluorescence intensity ratio decreases. NP tissue slices were incubated with a culture medium containing 10 *μ*M JC-1 for one hour at 37°C. After washing with PBS, the slices were immediately viewed using an inverted confocal laser scanning microscope, and one random image per disc was analyzed. The JC-1 red fluorescence intensity was analyzed using ImageJ software.

### 2.7. ROS Detection

Intracellular ROS generation was detected using dihydroethidium (MCE). Dihydroethidium, which penetrates the plasma membrane quite easily, is converted into ethidium bromide by superoxide anions and intercalates into DNA in the nucleus, emitting marked red fluorescence. NP slices were incubated with a culture medium containing 10 *μ*m dihydroethidium and 1 *μ*g/ml calcein AM for one hour at 37°C. After washing with PBS, the slices were immediately viewed using an inverted confocal laser scanning microscope, and one random image per disc was analyzed. The numbers of viable cells and dihydroethidium-positive cells were manually measured using ImageJ software to calculate the proportion of dihydroethidium-positive cells.

### 2.8. RNA Extraction and Real-Time Quantitative Polymerase Chain Reaction (RT-qPCR)

NP tissue was harvested on day 1 and day 7 for gene expression analysis. The cartilaginous endplates of each IVD were detached, and approximately 150 mg of NP tissue was collected. For RNA extraction, the tissue samples were digested with 2 mg/ml pronase for 1 hour at 37°C, flash frozen, pulverized in liquid nitrogen, and homogenized using a TissueLyser [27]. Total RNA extraction was performed using TRI Reagent (Molecular Research Center, Cincinnati, OH, USA), and then, 400 ng of RNA was converted to cDNA using a SuperScript VILO cDNA Synthesis Kit (Life Technologies, Carlsbad, CA). RT-qPCR was performed using PowerUp SYBR Green Master Mix (Thermo Fisher Scientific, USA) on a Real-Time System (Bio-Rad). Each reaction mixture was 10 *μ*l and contained 2 *μ*l of 5 ng/*μ*l cDNA, 5 *μ*l of 2x PowerUp SYBR Green Master Mix, 2 *μ*l of nuclease-free water, and 0.5 *μ*l each of 10 *μ*M forward and reverse primers. The following cycle conditions were applied: 50°C for 2 minutes and 95°C for 2 minutes followed by 44 cycles of 15 s at 95°C and 1 minute at 60°C. The specific primers used in this study were designed by using Primer 6.0 software (Applied Biosystems, Foster City, CA), and the sequences are provided in Table 1. Ribosomal protein lateral stalk subunit P0 (RPLP0) was used as a reference gene. The data were analyzed using the 2^-*ΔΔ*Ct^ algorithm.

### 2.9. Histology

NP tissues were fixed in 4% paraformaldehyde for 24 hours and dehydrated in graded sucrose solutions, after which 10 *μ*m thick sections were prepared. Immunofluorescence staining against CASPASE3 (1 : 400, Proteintech, China), BCL2 (1 : 200, Proteintech), BAX (1 : 400, Proteintech), MLKL (1 : 400, Invitrogen, CA, USA), MMP1 (1 : 200, Invitrogen), MMP3 (1 : 100, Proteintech), ADAMTS5 (1 : 200, Affinity, USA), and collagen II (1 : 200, Affinity) was performed. Briefly, the sections were permeabilized with 0.3% Triton X-100 for 30 minutes and then blocked with 5% bovine serum albumin and 0.1% Triton X-100 for 1 hour at room temperature. Subsequently, the sections were incubated with antibodies at 4°C overnight. The tissue sections were thoroughly washed with Tris-buffered saline with Tween-20 (TBST) and incubated with a Fluor-594-conjugated anti-rabbit secondary antibody (Jackson ImmunoResearch Inc., West Grove, PA, USA) at a 1 : 300 dilution for 1 hour at room temperature. Then, the sections were washed with TBST again, and the nuclei were counterstained with 4,6-diamidino-2-phenylindole (DAPI, Abcam, Germany) for 10 minutes.

Terminal deoxynucleotidyl transferase-mediated dUTP nick end labeling (TUNEL) was used to detect DNA fragmentation, which is known to be a characteristic of apoptosis. TUNEL staining was performed according to the instructions of a TUNEL Apoptosis Assay Kit (Dalian Meilun Biotech., Dalian, China), and the nuclei were counterstained with DAPI (Abcam) for 10 minutes. Images were visualized using an LSM 780 confocal microscope (Zeiss) with Zen Black software and analyzed using ImageJ.

After 0, 4, and 7 days of culture, IVDs were quickly fresh frozen, transected into 10 *μ*m thick sections and then fixed in 100% methanol. Safranin O (Sigma-Aldrich) and 0.02% Fast Green (Sigma-Aldrich) were used to show overall matrix organization, and Weigert's hematoxylin (Sigma-Aldrich) was used to show nuclear distribution. The stained sections were imaged with a digital pathology system (Kfbio, Ningbo, China). A semiquantitative scoring system was used to determine the degree of degeneration [18]. The histological grading criteria were based mainly on cleft patterns found in the IVDs, with scores ranging from 0 to 9.

### 2.10. Measurement of Oxidized Glutathione (GSSG) and Total Glutathione

GSSG and total glutathione were measured using a GSH (reduced glutathione) and GSSG Assay Kit (Beyotime Biotechnology, China). Briefly, NP tissues were pulverized in liquid nitrogen, homogenized in a buffer according to the instructions, and then centrifuged. To measure GSSG, GSH was blocked prior to the reaction with GSH reductase and NADPH. To measure total glutathione (GSSG + GSH), the supernatant was added to a buffer containing GSH reductase and NADPH. Five minutes later, dithionitrobenzoic acid (DTNB) was added, and the absorbance was measured at 412 nm.

### 2.11. Analysis of Released GAG

Cumulative release of GAG to the conditioned medium was measured using a modified 1,9-dimethylmethylene blue (DMMB) method [28]. The DMMB solution was prepared by dissolving 16 mg of DMMB (Sigma-Aldrich), 3.04 g of glycine (Sigma-Aldrich), and 2.37 g of NaCl in 1 L of distilled water (pH 3.0). Diluted conditioned medium (20 *μ*l) was mixed with 200 *μ*l of DMMB solution, and the absorbance was immediately measured at 535 nm. Serial dilutions of chondroitin 4-sulfate sodium salt (Aladdin, Shanghai, China) were used to generate the GAG standard reference curve.

### 2.12. Statistical Analysis

All statistical analyses were performed using SPSS 22.0 (IBM, Chicago, IL, USA). The Shapiro–Wilk normality test was performed to evaluate the normality of the data distribution. Comparisons between two groups were performed using Student's *t*-test for normally distributed data and Mann–Whitney *U*-tests for nonnormally distributed data. A difference was considered significant when the *P* value was <0.05.

## 3. Results

### 3.1. Presence of Mitochondrial ROS Accumulation and Mitochondrial Dysfunction in NP Cells after MS

Dihydroethidium staining was used to detect ROS production in NP cells at several time points after MS. MS significantly increased the ROS-positive cell proportion and remained at a stable high level over the first 12 hours (Figures 2(a) and 2(b)). Afterward, the proportion of ROS-positive cells decreased sharply and reached a low level by 48 hours. The proportion of ROS-positive cells remained stable in the physiological loading culture group. The mitochondrial electron transport inhibitor rotenone significantly reduced the proportion of ROS-positive cells immediately after MS (~78%, *P* < 0.01) (Figure 2(c)). The mitochondrial ROS scavenger MitoQ also significantly decreased the proportion of ROS-positive cells (~73%, *P* < 0.01).

JC-1 staining was used to monitor mitochondrial membrane potential in NP tissue immediately after MS. The NP cell mitochondrial membrane potential was significantly decreased in the MS group (Figures 2(d) and 2(e)). MitoQ pretreatment partially attenuated the depression of mitochondrial membrane potential. These results indicated that MS was able to directly induce mitochondrial dysfunction.

The GSSG/total glutathione ratio was calculated to further evaluate ROS levels in NP tissue. As shown in Figure 2(f), MS treatment increased the GSSG/total glutathione ratio, and this increase was alleviated by MitoQ pretreatment. In addition, RT-qPCR results showed that MitoQ significantly inhibited the mRNA expression of catalase (CAT) caused by MS (Figures 2(g) and 2(h)). These results demonstrated that the time-dependent ROS accumulation was mainly derived from the mitochondria after MS.

### 3.2. NP Cell Viability Change after MS

To explore the NP cell death mechanisms after MS, IVDs were cultivated and subsequently analyzed for cell viability at different time points. The application of MS to IVDs resulted in a dramatic time-dependent decrease in NP cell viability (Figures 3(a) and 3(b)). A small portion of NP cell death occurred immediately after MS, and cell viability remained stable during the first 12 hours ([CON vs. MS 0 hours]: 9.2%, *P* < 0.01; [MS 0 hours vs. MS 12 hours]: 1.9%, *P* > 0.05). More than 70% of NP cell death occurred within 12 to 48 hours after MS ([CON vs. MS 12 hours]: 11.1%, *P* < 0.05; [MS 12 hours vs. MS 48 hours]: 27.8%, *P* < 0.01). Cell viability reached a relatively stable status ([MS 48 hours vs. MS 72 hours]: 2.2%, *P* > 0.05) at 48 hours after MS application. Cell viability in the CON group remained stable at nearly 94% ([CON vs. CON 72 hours]: 1.8%, *P* > 0.05) after 72 hours in physiological loading culture. Thus, both the magnitude and the mechanism of cell death varied with time after MS.

The dramatic decrease in NP cell viability after 12 hours of MS suggested that, aside from necrosis that was directly caused by MS, programmed cell death was activated. For this reason, IVDs were pretreated with Z-VAD-FMK, Nec-1, or MitoQ for 2 hours and then subjected to MS. Cell viability analysis showed that inhibitor pretreatment significantly alleviated NP cell death (20% cell viability in the MitoQ group, *P* < 0.05; 15.82% cell viability in the Z-VAD-FMK group, *P* < 0.05; 13.12% cell viability in the Nec-1 group, *P* < 0.05) with respect to the MS group (Figure 3(c)).

### 3.3. Programmed Cell Death-Associated Marker Changes in NP Tissue after MS

We further investigated the relative changes in apoptosis indicator genes (CASPASE3, BCL2, and BAX) and necroptosis indicator genes (RIP1, RIP3, and MLKL) (Figures 4(a)–4(f)). The mRNA expression levels of apoptosis and necroptosis genes were significantly increased at 12 hours after MS, and MitoQ pretreatment alleviated some of these changes (CASPASE3, RIP1, RIP3, and MLKL). In line with the mRNA expression results, the results of immunofluorescence staining showed that apoptosis (CASPASE3, BAX, and BAX/BCL2 radio) and necroptosis (MLKL) were significantly increased at 12 hours after MS (Figures 4(g)–4(j) and 4(m)). MitoQ pretreatment significantly suppressed the expression of the programmed cell death-related markers MLKL, CASPASE3, and BAX and elevated the expression of BCL2. In addition, TUNEL staining indicated that MitoQ remarkably reversed the NP cell apoptosis caused by MS (*P* < 0.01) (Figures 4(k) and 4(l)).

To determine whether MS has a long-lasting impact on NP cell programmed death, the mRNA/protein levels of apoptosis and necroptosis genes and proteins were measured in the 7-day MS group. The levels of these markers were not significantly different between the 7-day MS group and the 7-day CON group (Figures 4(a)–4(j) and 4(m)). TUNEL staining indicated that there was no significant difference in the level of apoptosis between these two groups (Figures 4(k) and 4(l)).

### 3.4. Metabolic Dysregulation in NP Tissue after MS

NP tissue from both the MS group and the CON group was harvested for metabolic analysis at 12 hours and 7 days after MS. Compared with the CON group, the MS group exhibited upregulated catabolic gene (MMP1, MMP3, and ADAMTS5) expression levels and downregulated collagen type II alpha 1 (COL2A1) expression levels 12 hours after MS (Figures 5(a)–5(f)). The immunofluorescence staining results further confirmed the above changes (Figures 5(g)–5(j)). MitoQ pretreatment partly alleviated the MS-induced metabolic dysregulation.

To further investigate the extent of metabolic dysregulation, we analyzed cumulative GAG release using the DMMB method. The conditioned medium was collected daily after free-swelling culture. The value measured on day 1 was used as a baseline for normalization. MS significantly increased the cumulative GAG release on day 7. MitoQ pretreatment partially prevented GAG loss (Figure 5(k)).

### 3.5. Dynamic Compressive Stiffness and Morphology of IVDs

On the first day after MS, the changes in dynamic compressive stiffness did not significantly differ among the CON, MS, and MitoQ + MS groups (Figure 6(c)). Compared with those in the CON group, the IVDs in the MS group exhibited significantly lower stiffness on day 7, but this difference was attenuated by MitoQ (Figure 6(d)). These results indicated that MS reduced the stiffness of IVDs partly through mitochondrial ROS.

We then evaluated the morphology of IVDs by Safranin O/Fast Green and hematoxylin staining. Seven days after MS application, the MS group had significantly higher degeneration scores than the CON group. Moreover, there were no significant differences in degeneration scores between day 4 and day 7 after MS application. In MitoQ-pretreated IVDs, the degeneration scores were significantly reduced (Figures 6(e) and 6(f)).

## 4. Discussion

MS has been identified as a significant risk factor for the onset and progression of DDD [27]. Numerous reports have suggested that sophisticated molecular cascades are involved in the pathophysiology of MS-induced DDD [29, 30]. In the current study, we attempted to address the interplay between mitochondrial ROS and DDD in an IVD organ culture model by using a custom-made universal mechanical tester. We obtained evidence that multiple modes of cell death are involved in MS-induced NP cell death, with mitochondrial ROS-orchestrated programmed cell death playing a critical role. Our data suggest that mitochondrial ROS are the primary sources of oxidants in IVDs after MS. In addition, we found that MS-induced ECM degeneration is mediated, at least in part, by mitochondrial ROS. Furthermore, we found that MS alters metabolic and programmed cell death-related marker expression levels at early time points.

ROS, as pleiotropic pathophysiological signaling agents, are generated from diverse intracellular sources, including cytosolic membrane NADPH oxidase, mitochondrial respiratory complexes, xanthine oxidase, and uncoupled nitric oxide synthase [31]. Accumulating evidence suggests that ROS play a crucial role in the onset and exacerbation of DDD [32]. Although a number of studies have suggested that mitochondrial-derived ROS participate in DDD, no studies have investigated the primary sources of ROS in NP cells after MS. MitoQ is a mitochondrial-targeted ROS scavenger that has been shown in numerous studies to alleviate oxidative damage and decrease mitochondrial ROS levels [33]. We used MitoQ in our research to elucidate the importance of mitochondrial ROS in MS-induced cell death and ECM degradation. We also used rotenone to inhibit mitochondrial respiratory chain complex I. Rotenone pretreatment significantly and immediately inhibited ROS production after MS. In addition, the mitochondrial-targeted antioxidant MitoQ attenuated large-scale MS-induced ROS production. Thus, the data suggested that mitochondrial ROS were the main sources of oxidants in our model system. We also studied the time course of ROS generation. The proportion of ROS-positive cells reached a high level at the earliest observation time point. Long-term follow-up revealed that the proportion of positive cells remained stable from 0 to 12 hours but decreased sharply by 24 hours and reached a relatively low level at 48 hours after MS. These data indicate that ROS-related pathological changes may be limited to the early stage after MS.

In ex vivo studies using bovine IVD whole-organ culture models, MS has been found to reduce NP cell viability [34]. However, the NP cell death mode and time course have remained largely unknown. Live/dead cell analysis of IVDs revealed that cell viability remained steady during the first 12 hours after MS, except that a few cells were lost immediately after MS, and that subsequent large-scale cell death occurred at 24 hours. The acute cell loss might have resulted from necrotic cell death induced by MS. The later occurrence of large-scale cell death suggested that, in addition to necrosis, programmed cell death was initiated.

In vitro experiments using a variety of cell culture compression apparatuses have shown that MS to NP cells induces apoptosis and necroptosis [15]. However, previous reports have focused mainly on short-term changes in the cell death mode, and there have been no reports about the long-term effects of MS on NP cells. To our knowledge, this is the first study to investigate the changes in programmed death after MS injury at early time points (12 hours) and long-term time points (7 days). In line with previous studies, our study demonstrated that necroptosis and apoptosis occurred in the IVD organ culture model in response to MS at early time points. However, necroptosis- and apoptosis-associated markers returned to normal levels by day 7 after force application. These data demonstrated that the influence of MS on NP cell viability was confined to a relatively short period.

The time course of NP cell death was consistent with the kinetics of mitochondrial ROS in this model, which peaked and then remained stable during the first 12 hours before decreasing to a relatively low level by 48 hours after MS. It is reasonable to suppose that mitochondrial ROS were partly responsible for the induction of necroptosis and apoptosis. In this study, MitoQ pretreatment significantly improved cell viability and partially restored necroptosis- and apoptosis-associated marker levels in the IVD model. Therefore, the results indicated that MS induced apoptosis and necroptosis via mitochondrial ROS in NP cells.

Similar to a number of previous studies, our study revealed that MS increased catabolic gene expression and ECM degeneration [35]. In the present study, using an ex vivo bovine IVD organ culture model, we found that MitoQ pretreatment attenuated the ECM degeneration and reduced catabolic marker expression. Based on the previously reported deleterious effects of ROS on the expression of catabolic markers and ECM integrity, these findings indicate that increased mitochondrial ROS levels are partly responsible for MS-induced degenerative changes in the disc NP region. As a previous study failed to provoke matrix degradation via catabolic molecules in bovine IVDs, further investigation is needed to explore the potential molecular mechanisms responsible for mitochondrial ROS-mediated NP tissue degeneration [36].

There were several limitations of our study. First, the ex vivo IVD organ model used in our study was subjected to acute compressive MS. Whether the research findings can be applied to complex physiological MS needs further investigation. Second, we confirmed that mitochondrial ROS are partly responsible for the induction of programmed NP cell death after MS, but we did not elucidate the precise molecular mechanisms. Third, the mitochondrial ROS elevation discussed in our study may represent only a small proportion of the mitochondrial dysfunction mechanisms at play. More intricate mechanisms of mitochondrial dysfunction in DDD should be further investigated in future studies.

## 5. Conclusions

The data demonstrate that ROS induce programmed NP cell death and ECM degradation at early time points after MS. These accumulated ROS are derived mainly from mitochondria. These findings suggest that the use of mitochondrial-targeted antioxidants immediately after MS may be a promising method to prevent the onset or progression of DDD. Our results also provide novel insight into the pathological mechanism of DDD.

## Figures and Tables

**Figure 1:** (a) Bioreactor and custom-designed chamber for physiological loading and the universal mechanical tester for MS on bovine IVDs. (b) Flow chart describing the study design.

**Figure 2:** MS induced large-scale mitochondrial ROS generation and mitochondrial dysfunction. (a) Typical confocal images showing the viable cells (green) and ROS-positive cells (red) in the CON group and the MS group at 0 hours after MS. (b) Percentages of ROS-positive cells measured in the CON group and the MS group at different time points. (c) Rotenone and MitoQ pretreatment reduced the percentage of ROS-positive cells. (d) Typical confocal images of JC-1 staining showing the red fluorescence of JC-1 aggregates and the green signal of JC-1 monomers at 0 hours after MS. (e) Quantification of the mitochondrial membrane potential (ratio of red to green fluorescence) in the CON, MS, and MitoQ pretreatment groups. (f) The relative ratio of GSSG to total glutathione was measured at 12 hours after MS. (g, h) Quantification of SOD2 and CAT mRNA levels at 12 hours after MS. Scale bars, 50 *μ*m and 5 *μ*m (inset). The values are expressed as the means ± SEMs. *n* = 3, ^∗^*P* < 0.05, and ^∗∗^*P* < 0.01.

**Figure 3:** The time course of MS-induced NP cell death. (a) Typical confocal images showing the dead cells (red) and viable cells (green) after MS at different time points (0 hours, 6 hours, 12 hours, 24 hours, 48 hours, and 72 hours). Scale bars, 50 *μ*m. (b) Quantification of the ratio of viable cells to total cells in the CON group and the MS group at different time points. (c) Quantification of the ratio of viable cells to total cells in the MitoQ, Nec-1, and Z-VAD pretreatment groups. Values are expressed as the means ± SEM. *n* = 3, ^∗^*P* < 0.05, and ^∗∗^*P* < 0.01.

**Figure 4:** MS induced programmed NP cell death via mitochondrial ROS. (a–f) Necroptosis- and apoptosis-related gene expression in NP tissue was examined using RT-qPCR. The gene expression levels in the MS group and the MitoQ + MS group are expressed relative to those in the CON group at 12 hours after MS. The expression levels in the MS 7-day group were similar to those in the CON 7-day group. *n* = 3. (g–j) Necroptosis- and apoptosis-related markers in NP tissue were examined using immunohistochemical staining. Scale bars, 50 *μ*m and 5 *μ*m (inset). *n* = 3. (k, l) Apoptotic NP cells were examined using TUNEL staining, and the percentage of positive cells was quantified. Scale bars, 50 *μ*m. *n* = 3. (m) Quantification analysis of the Bax/Bcl-2 immunohistochemical staining ratio. The data are expressed as the means ± SEMs. ^∗^*P* < 0.05 and ^∗∗^*P* < 0.01.

**Figure 5:** Mitochondrial ROS participated in MS-mediated metabolic dysregulation. Gene expression was analyzed by RT-qPCR for (a) MMP1, (b) MMP3, (c) MMP13, (d) ADAMTS4, (e) ADAMTS5, and (f) COL2A1. The gene expression levels in the MS group and the MitoQ + MS group are expressed relative to those in the CON group at 12 hours after MS. The expression levels in the MS 7-day group were similar to those in the CON 7-day group. The data are expressed as the means ± SEMs. *n* = 5. (g–j) Anabolic-related markers and collagen II in NP tissue were examined using immunohistochemical staining. Scale bars, 50 *μ*m and 5 *μ*m (inset). *n* = 3. (k) Cumulative release of GAG into a culture medium. *n* = 3. The data are expressed as the means ± SEMs. ^∗^*P* < 0.05 and ^∗∗^*P* < 0.01.

**Figure 6:** Mitochondrial ROS participated in MS-induced IVD dynamic compressive stiffness reduction and morphological degenerative changes. (a) Representative strain curves of the IVDs during stiffness gauging at a single time point. (b) Representative stress curves of the IVDs during stiffness gauging at a single time point. (c, d) Dynamic compressive stiffness measured on day 1 after overnight swelling (the day after dissection), on day 2 after overnight swelling (the day after MS), and on day 7 after overnight swelling recovery. The data were normalized to the levels on day 1 after overnight swelling. (e) The morphology of the IVDs was evaluated by Safranin O/Fast Green staining. Scale bars, 625 *μ*m. (f) Degeneration scores based on Safranin O/Fast Green staining. The data are expressed as the means ± SEMs. *n* = 3, ^∗^*P* < 0.05, and ^∗∗^*P* < 0.01.

**Table 1:** Primers used for RT-qPCR.

ADAMSTS4	F:5′-TACCGAGGGACTGAACTCCACATC-3′ R:5′-GGAATGCCGCCATCTTGTCATCT-3′

ADAMSTS5	F:5′-TGTGCGGTGATTGAAGACGATGG-3′ R:5′-TGCTGGTGAGGATGGAAGACATTAAG-3′

BAX	F:5′-TTTGCTTCAGGGTTTCATCCAGGATC-3′ R:5′-AGACACTCGCTCAGCTTCTTGGT-3′

BCL2	F:5′-TGTGGATGACCGAGTACCTGAAC-3′ R:5′-GAGACAGCCAGGAGAAATCAAACAG-3′

CASPASE3	F:5′-CGCATATTCTACAGCACCTGGTTAC-3′ R:5′-AGCATCTCACAAAGAGCCTGGAT-3′

CAT	F:5′-TCAACAGTGCCAACGATGACAATG-3′ R:5′-GATGCGGGAGCCATATTCAGGAT-3′

COL2A1	F:5′-GAGCAGCAAGAGCAAGGACAAGA-3′ R:5′-GCAGTGGTAGGTGATGTTCTGAGAG-3′

MLKL	F:5′-CAGACTTCCATCAGCCGACAAACTA-3′ R:5′-ATCTCCCAGAGGACAATTCCAAAGC-3′

MMP1	F:5′-CCAGACCTGTCAAGAGCAGATGT-3′ R:5′-ATGAGCGTCTCCTCCGATACCT-3′

MMP3	F:5′-AACCTTCCGATTCTGCTGTTGCTA-3′ R:5′-GCTTGCGTATCACCTCCAGAGT-3′

MMP13	F:5′-AGACAAATGTGACCCTTCC-3′ R:5′-ATAGGCGGCATCAATACG-3′

RIPK1	F:5′-CTCGCTTACCCTGGTGTGATGA-3′ R:5′-TGATGGCAAGGAGGTGAATGGA-3′

RIPK3	F:5′-TCAAGCCCTCCAATGTCCTACTAGA-3′ R:5′-ACTGTGAGCCTCCCTGAAATGTG-3′

RPLP0	F:5′-CACGCTGCTGAACATGCTGAAC-3′ R:5′-AGGCACACGCTGGCAACATT-3′

SOD2	F:5′-TCTTCTGGACAAATCTGAGCCCTA-3′ R:5′-TCCTGGTTAGAACAAGCAGCAATC-3′

## Data Availability

The data used to support the findings of this study are available from the corresponding author upon request.
